# Role of the PEBP4 protein in the development and metastasis of gastric cancer

This article has been retracted.

**DOI:** 10.18632/oncotarget.15255

**Published:** 2017-02-10

**Authors:** Zijian Wu, Bin Liu, Xuemin Zheng, Huijing Hou, Ying Li

**Affiliations:** ^1^ Tianjin Key Laboratory of Food Biotechnology, College of Biotechnology and Food Science, Tianjin University of Commerce, China; ^2^ Tianjin Institute of Pharmaceutical Research, China; ^3^ Tianjin Neurological Institute, Tianjin Medical University General Hospital, China

**Keywords:** gastric cancer, PEBP4, cancer immigration, cancer invasion

## Abstract

Phosphatidylethanolamine-binding protein 4 (PEBP4) has previously been reported to be upregulated in various cancers. However, the physiological functions of PEBP4 in gastric cancer are still unknown. Aiming to clarify the properties and role of PEBP4 in the development and invasion of gastric cancer, we performed several biological assays and a knockdown assay. The expression level of PEBP4 was shown to be significantly upregulated in gastric cancer tissue samples, and knockdown of the expression of PEBP4 induced significant inhibitory effects on cell proliferation, migration and invasiveness. In addition, it was demonstrated that PEBP4 was associated with the development and invasion of gastric cancer cells through activation of the PI3K/Akt signaling pathway. Our findings supported the hypothesis that PEBP4 might be a novel potential drug target for the treatment of gastric cancer.

## INTRODUCTION

Gastric cancer is one of the main contributors to cancer-related mortality worldwide [1]. Despite recent developments in early diagnosis and other novel therapeutic strategies, the median survival time for advanced gastric cancer patients has still remained at approximately 7 months [2, 3]. Thus, investigations into the molecular mechanisms of invasion and metastasis of gastric cancer seek to contribute to the development of a novel and effective drug target.

Phosphatidylethanolamine-binding protein 4 (PEBP4) is a member of the PEBP family, which shares a similar domain consisting of a C-terminal large β-sheet flanked by smaller β-sheets and 2 α-helices [4]. It has been reported that PEBP4 plays important roles in multiple biological processes, including the synthesis of the cell membrane, myoblast differentiation, neural development and tumorigenesis [5–8]. Recently, the upregulation of PEBP4 was reported to be associated with the proliferation, invasion and drug resistance of tumor cells [9, 10]. However, direct evidence for the role of PEBP4 in cancer development and invasion is still lacking. In this study, we silenced the expression of PEBP4 by specific siRNA in gastric cancer cell lines and investigated the effects of PEBP4 on cell proliferation, migration and invasion. Our results show that the effects of PEBP4 on the tumorigenesis and metastasis of gastric cancer depend on the dysregulation of the PI3K/Akt signaling pathway.

## RESULTS

### PEBP4 is highly expressed in gastric cancer tissue and cell lines

To explore the potential role of PEBP4 in the tumorigenesis of gastric cancer, the mRNA levels of PEBP4 were studied in gastric cancer tissue samples and the corresponding adjacent normal tissue samples from 11 patients using RT-qPCR. The mRNA levels of PEBP4 in human gastric cancer tissue were significantly higher than those in the adjacent normal gastric tissue, as shown in Figure 1A. The western blot results showed that the expression level of the PEBP4 protein was markedly higher in human gastric cancer tissue samples than in normal gastric tissue samples (Figure 1B). Similarly, the mRNA and protein expression levels of PEBP4 were also increased in gastric cancer cell lines (Figure 1C and 1D).

**Figure 1:** Expression of PEBP4 was upregulated in gastric cancer tissue samples and cell lines **(Panel A)** QRT-PCR analysis of PEBP4 mRNA in 11 human gastric cancer tissue samples and paired adjacent normal gastric tissue samples. PEBP4 mRNA levels in human gastric cancer tissue were markedly higher than those in normal gastric tissue. **(Panel B)** Western blot analysis of PEBP4 protein in gastric cancer tissue and normal gastric tissue; *P<0.05 compared with the normal gastric tissue. **(Panel C)** The representative mRNA expression of PEBP4 in human gastric cancer cell lines. **(Panel D)** The representative western blot image of the PEBP4 protein in human gastric cancer cell lines. Data are expressed as the mean ± SD. Experiments were performed in triplicate. *P<0.05 compared with the GES-1 cells.

### Knockdown of PEBP4 inhibited the proliferation, migration and invasion of gastric cancer cells

To clarify the role of PEBP4 on cell proliferation, migration and invasion, the TSGH and AGS cells were transfected with siRNA-PEBP4 or siRNA-control. The western blot results demonstrated a remarkable downregulation of PEBP4 expression in TSGH and AGS cells (Figure 2A). The results of the cell proliferation assay indicated that knockdown of PEBP4 greatly suppressed the proliferation of both types of cells in a time-dependent manner (Figure 2B). Additionally, knockdown of PEBP4 resulted in a remarkable reduction in tumor cell migration and invasion (Figure 3).

**Figure 2:** Knockdown of PEBP4 inhibited the proliferation of gastric cancer cells **(Panel A)** Western blot of analysis of PEBP4 in TSGH and AGS cells. **(Panel B)** Proliferation of TSGH and AGS cells was detected using the BrdU assay. TSGH and AGS cells were transfected with siRNA against PEBP4 and scrambled siRNA for 24 h. Data are expressed as the mean ± SD. Experiments were performed in triplicate. *P<0.05 compared with the scramble group.

**Figure 3:** Knockdown of PEBP4 inhibited the migration and invasion of gastric cancer cells **(Panel A)** The migration of the indicated cells was evaluated by a Transwell assay; cells that passed through the Matrigel membrane after 24 h were counted in five representative microscopic fields. **(Panel B)** The invasiveness of the indicated cells was evaluated by a Matrigel-coated Transwell assay; cells that passed through the Matrigel membrane after 24 h were counted in five representative microscopic fields. TSGH and AGS cells were transfected with siRNA against PEBP4 and scrambled siRNA for 24 h. Data are expressed as the mean ± SD. Experiments were performed in triplicate. *P<0.05 compared with the scramble group.

Interestingly, knockdown of PEBP4 was found to retard the epithelial-mesenchymal transition (EMT) phenotype in gastric cancer cells. The RT-qPCR results indicated that knockdown of PEBP4 resulted in a significant increase in the mRNA levels of E-cadherin and a decrease in N-cadherin in TSGH cells (Figure 4A) and AGS cells (Figure 4B). Similarly, the western blot results also suggested an inhibitory effect on the EMT in gastric tumor cells upon knockdown of PEBP4 (Figure 4C).

**Figure 4:** Knockdown of PEBP4 inhibited the epithelial-mesenchymal transition (EMT) phenotype in gastric cancer cells **(Panel A, B)** Total RNA was isolated from the indicated cells; the expression of E-cadherin and N-cadherin was analyzed using RT-qPCR. **(Panel C)** Total protein was isolated form the indicated cells, and EMT markers were measured using western blot analysis. TSGH and AGS cells were transfected with siRNA against PEBP4 and scrambled siRNA for 24 h. Data are expressed as the mean ± SD. Experiments were performed in triplicate. *P<0.05 compared with the scramble group.

It was observed that knockdown of PEBP4 greatly inhibited the phosphorylation of PI3K and Akt, suggesting that PEBP4 might exert its physiological functions *via* modulation of the PI3K/Akt signaling pathway (Figure 5).

**Figure 5:** Knockdown of PEBP4 inhibited the activation of the PI3K/Akt signaling pathway The levels of phosphorylated PI3K, total PI3K, phosphorylated Akt, and total Akt were analyzed using western blot analysis. TSGH cells were transfected with siRNA against PEBP4 and scrambled siRNA for 30 min.

## DISCUSSION

PEBP4 has been reported to be involved in the tumor development and metastasis of various cancers [11]. For example, PEBP4 has been reported to be upregulated in pancreatic ductal adenocarcinoma (PDAC), and knockdown of PEBP4 has been shown to result in the attenuation of cancer cell growth, migration, and metastasis of PDAC cancer cells [10]. In lung cancer, PEBP4 is capable of enhancing the cell proliferation and invasion ability [12]. Liu et al. reported that PEBP4 in colorectal cancer tissues was markedly increased and the downregulation of PEBP4 significantly reduced the migration of colorectal cancer cells in a Transwell chamber [13].

In the present study, PEBP4 was first demonstrated to be upregulated in gastric cancer tissue samples and cell lines. Knockdown of PEBP4 inhibited cell proliferation, migration and invasiveness. EMT is an important process during tumor development, characterized by reduced intercellular adhesion and enhanced motility of epithelial cells [14]. As one of the markers of EMT, the measurement of the levels of E-cadherin and N-cadherin was a crucial approach to investigate the EMT phenotype and then evaluate tumor invasion [15]. In the present study, knockdown of PEBP4 was found to remarkably increase the expression of E-cadherin and decrease the expression of N-cadherin in TSGH and AGS cells. The results suggested that knockdown of PEBP4 retarded the EMT process in gastric cancer cells, which might have contributed to the inhibitory effect of the siRNA-PEBP4 on tumor migration and invasion.

The PI3K/Akt pathway was determined to be associated with proliferation, metastasis, apoptosis and EMT in gastric cancer [16–21]. Treatment of gastric cancer cells with a PI3K/Akt kinase inhibitor significantly retarded the EMT phenotype by inhibiting bone morphogenetic protein (BMP)-2 [22, 23]. PEBP4 was previously found to be crucial for the phosphorylation of Akt at serine^473^ [10]. Additionally, the silencing of hPEBP4 in TRAIL-resistant human prostate cancer cells inhibited Akt activation [24]. In this study, it was also found that knockdown of PEBP4 markedly inhibited the phosphorylation of PI3K and Akt in gastric cancer cells.

Together, the results in this study supported the hypothesis that knockdown of PEBP4 inhibits cell invasion and EMT through suppressing the PI3K/Akt signaling pathway. These results suggest that PEBP4 might be potential drug target for the treatment of gastric cancer.

## MATERIALS AND METHODS

### Tissue sample collection

Gastric cancer tissue samples were obtained from 11 patients undergoing surgical treatment at the Department of Oncology, Tianjin Medical University General Hospital (China), during the period from 2014 to 2015 (average age=59.6). All of the patients received primary treatments by surgery, chemotherapy or hormone therapy. Healthy tissue samples were from non-pathologic areas distant from the tumors in surgical specimens. The fresh tissue specimens were immediately snap-frozen and stored in liquid nitrogen until use. The protocol for the use of patient samples was approved by the Biomedical Ethics Committee of the Tianjin Medical University General Hospital.

### Cell culture

Three human gastric cancer cell lines (TSGH, N87 and AGS) and a normal gastric mucosal epithelial cell line (GES-1) were purchased from the American Type Culture Collection (ATCC, Manassas, VA). The cells were cultured in RPMI 1640 medium (Invitrogen, Carlsbad, CA, USA) supplemented with 10% fetal bovine serum (FBS; Gibco, Rockville, MD), penicillin (100 units/ml), streptomycin (100 μg/ml), L-glutamine (2 mM), and sodium pyruvate (1 mM) in a humidified incubator with 5% CO_2_ at 37°C.

### siRNA knockdown of PEBP4

Small interfering RNA (siRNA) for PEBP4 knockdown was designed and synthesized by Guangzhou RiboBio (Guangzhou, China), and the primer sequences for PEBP4 were: 5’-ACTGGGTCTCATGATGGTGG-3’, and 5’-CTCCATCCAGGAGGTGATCT-3’; and the primer sequences for β-actin were: 5’-TTAGTTGCGTTACACCCTTTC-3’ and 5’-ACCTTCACCGTTCCAGTTT-3’. For transfection, the cells were seeded in a 24-well plate for 24 h until they reached 50% confluence. The cells were transfected with 2 μl (20 μM) siRNA using a Lipofectamine™ 2000 reagent (Invitrogen, Carlsbad, CA) according to the manufacturer's instructions, and then cells were incubated at 37°C in a CO_2_ incubator for 48 h before the siRNA knockdown assay.

### Cell proliferation assay

Cells were transfected with siRNA-PEBP4 and siRNA control. After 24 h of serum starvation, the cells were incubated with BrdU solution at 37°C for 24 or 48 h using the cell proliferation ELISA BrdU kit (Takara Biotechnology, Dalian, China). The amount of BrdU was measured at 450 nm by a microplate reader (Bio-Rad, Hercules, CA, USA).

### Cell migration and invasion assays

The invasion and migration of gastric cancer cells upon downregulation of PEBP4 were analyzed by a Transwell chamber (Corning Costar Corp., Cambridge, MA, USA) assay. The TSGH and AGS cells treated with siRNA-PEBP4 or siRNA-control (1×10^5^ cells/ml) were added to the upper chamber. The lower chamber of the Transwell was filled with 500 μl DMEM containing 10% FBS as a chemo-attractant. After 24 h incubation, cells on the surface of the upper chamber were removed by scraping with a cotton swab. The migrated cells on the lower surface of the chamber were stained with 0.1% crystal violet (Sigma, MO) and counted. These experiments were repeated three times.

For the invasion assay, cells were seeded onto a Matrigel-coated membrane matrix (BD Biosciences, Bedford, MA, USA) in a 24-well culture plate for 24 h after transfection. The cells that did not invade through the pores were carefully wiped with cotton wool. Then, cells located on the lower surface of the chamber were stained with 0.1% crystal violet (Sigma, MO) and counted. These experiments were repeated three times.

### RNA extraction and quantification using reverse transcription polymerase chain reaction (RT-qPCR)

Total RNA was extracted from gastric cancer tissue and cells using Trizol reagent (Abcam, Cambridge, UK) according to the manufacturer's instructions. cDNA was prepared using the EasyScript First-Strand cDNA Synthesis SuperMix kit (Invitrogen, Carlsbad, CA, USA). PCR amplification was performed using the following primers: PEBP4, 5’-ACTGGGTCTCATGATGGTGG-3’ (sense), and 5’-CTCCATCCAGGAGGTGATCT-3’ (antisense); and β-actin, 5’-TTAGTTGCGTTACACCCTTTC-3’ (sense) and 5’-ACCTTCACCGTTCCAGTTT-3’ (antisense). The RT-qPCR conditions included an initial denaturation step at 94°C for 2 min, followed by 35 cycles of 94°C for 30 s, 56°C for 30 s, and 72°C for 2 min, and a final elongation step at 72°C for 10 min.

### Western blot

The expression levels of desired proteins extracted from gastric cancer tissues were analyzed using a standard western blot assay. Proteins were transferred onto polyvinylidene fluoride (PVDF) membranes (Millipore, Boston, MA, USA). The treated membrane was incubated in primary antibodies (anti-PEBP4, anti-E-cadherin, anti-N-cadherin, anti-PI3K, anti-p-PI3K, anti-p-Akt, anti-Akt and anti-GAPDH) (Santa Cruz Biotechnology, Santa Cruz, CA, USA) at 4°C overnight. Membranes were then incubated with horseradish peroxidase-conjugated secondary antibodies. The protein concentrations were visualized and calculated by chemiluminescence (Boehringer Mannheim GmbH, Mannheim, Germany) and BandScan 5.0 software.

### Statistical analysis

All results are reported as the means ± SD. For statistical analysis, a Student's t-test was used for the comparison of two groups, and a one-way ANOVA was used for multiple comparisons. *P*<0.05 was considered to be significant.
